# *Solanum tuberosum* Leaf Extract Templated Synthesis of Co_3_O_4_ Nanoparticles for Electrochemical Sensor and Antibacterial Applications

This article has been retracted.

**DOI:** 10.1155/2022/8440756

**Published:** 2022-03-08

**Authors:** Eneyew Tilahun Bekele, H. C. Ananda Murthy, Dhanalakshmi Muniswamy, Yeshaneh Adimasu Lemenh, Minale Shegaw Shume, Gezahegn Tadesse Ayanie, Avvaru Praveen Kumar, C. R. Ravikumar, R. Balachandran, Arpita Roy

**Affiliations:** ^1^Department of Applied Chemistry, School of Applied Natural Science, Adama Science and Technology University, P O Box 1888, Adama, Ethiopia; ^2^Department of Physics, Government Science College (Nrupathunga University), Bengaluru 560 001, India; ^3^Department of Applied Biology, School of Applied Natural Science, Adama Science and Technology University, P O Box 1888, Adama, Ethiopia; ^4^Department of Applied Physics, School of Applied Natural Science, Adama Science and Technology University, P O Box 1888, Adama, Ethiopia; ^5^Research Centre, Department of Science, East-West Institute of Technology, Bangalore 560091, India; ^6^School of Electrical Engineering and Computing, Adama Science and Technology University, P O Box 1888, Adama, Ethiopia; ^7^Department of Biotechnology, School of Engineering & Technology, Sharda University, Greater Noida, India

## Abstract

Green synthesis of metal oxide nanoparticles (NPs) is a viable alternative methodology because of cost-effective and availability of environmentally friendly templates for desired application, which has attracted the attention of researchers in recent years. In the present study, Co_3_O_4_ NPs were synthesized in various volume ratios in the presence of *Solanum tuberosum* leaf extract as a template. The synthesized Co_3_O_4_ NPs were characterized by X-ray diffraction (XRD), scanning electron microscopy-energy dispersive X-ray spectroscopy (SEM-EDX), transmission electron microscopy (TEM), high resolution transmission electron microscopy (HRTEM), surface area electron diffraction (SAED), UV-Vis diffuse reflectance spectroscopy (UV-DRS), and Fourier transform infrared (FTIR) spectroscopy. XRD analysis found that the average crystalline sizes for the 1 : 2, 1 : 1, and 2 : 1 volume ratios was 25.83, 21.05, and 27.98 nm, respectively. SEM-EDX and TEM analyses suggest that the green-synthesized Co_3_O_4_ NPs are spherical in shape without the presence of impurities. The band gap *E*_*g*_ values of the 1 : 2, 1 : 1, and 2 : 1 volume ratios of Co_3_O_4_ NPs were found to be 1.83, 1.77, and 2.19 eV, respectively. FTIR analysis confirmed the presence of various bioactive ingredients within the leaf extract of *Solanum tuberosum*. Co_3_O_4_ NPs-modified electrodes showed better sensing capability towards ascorbic acid and citric acid due to enhanced electron transfer kinetics. Among three volume ratios (1 : 2, 1 : 1, and 2 : 1) of Co_3_O_4_ nanoelectrodes, 1 : 1 and 2 : 1 were identified as the best performing nanoelectrodes. This is possibly due to the high catalytic behavior and the more homogenized surface structure. Co_3_O_4_ (1 : 2) nanodrug showed the enhanced antibacterial activity (16 mm) towards *S. aureus* which is attributed to the formation of enhanced reactive oxygen species (ROS).

## 1. Introduction

Ascorbic acid abbreviated as AA, commonly known as vitamin C, is one of the most imperative nutrients existing in the extracellular fluid of the human central nervous system and found to be an effective antioxidant species, which is used for the treatment of many health problems of human beings [1]. AA is a crucial water-soluble vitamin, which is not synthesized directly by the human body, instead present naturally within various diet sources such as lemon, orange, tomato, pepper, leafy vegetables, and drinks. By nature, AA plays a pillar role in various areas such as in clinical pharmacy, food industry, industrial and environmental procedures, cosmetic, and biomedical chemistry [2]. Moreover, AA acts as an antioxidant to prevent oxidation of food sources, food additives, neurotransmitter within the brain, and also as an enzyme cofactor [3].

Similarly, citric acid (CA) is also known as a natural weak acid, and it plays a vital role in everyday human activities such as the production of vinegar, ester, polymeric-based materials, reduction of blood sugar, to lose excessive weight, to cure and treat soreness and congestion of throat, for acid level regulation, to remove dead skin cells, and as a chelating agent [4]. Citrate anion exists in the form of anhydrous or monohydrate and is naturally present in several foods and serves as a nutrient in the human body. In particular, citrate ion is widely used in the pharmaceutical industry as an anticoagulant agent to stop accidental blood clotting and in the food industry as a preservative across the broad spectrum of foods and various beverage products. Since, citrate especially in urine is considered to inhibit the crystallization of the content of calcium salt leading to nephrolithiasis and hypocitraturia [5].

The intake of both AA and CA contents decreases below or above the standard and recommended amount results in severe sickness and general disorderness [6]. So, now-a-days, numerous electrochemical and analytical determination protocols for the determination of AA and CA have been developed such as titration, chromatography, colorimetry, fluorescence, spectrophotometry, capillary electrophoresis, voltammetry, fluorometry, spectrometry, chemiluminescence, and enzymatic approaches [2, 7]. However, it has been reported that these analytical approaches are relatively complicated, expensive, unsuitable, time-consuming, less sensitive, and less selective. The various electrochemical protocols used for the detection and measurement of AA and CA concentration have been become much attractive as compared to the numerous conventional analytical methods. Although the electrochemical methods of AA and CA detection are best compared to the counter components, uncoated bare electrodes still have some limitations and failures. Therefore, to overcome the limitations and shortcoming of those bare electrodes, a number of advanced techniques with many advantages such as high surface area, good stability and fast electron transfer kinetics, simple preparation, low cost, high specificity, and improved electrochemical and electrical properties have received extensive researcher's attention [8].

One of the global and current research concerns related to health and the natural environment is found to be the increasing of antimicrobial resistance against chemically synthesized and fabricated antibiotics. Majority of the various classifications of pathogens that could have been cured in the past are now becoming untreatable [9]. A rapid increase in the development and improvement of new antibacterial inorganic and organic drugs has been observed due to the high prevalence of antibiotic resistant infection which is a serious problem worldwide [10]. To overcome those problems worldwide, the search, design, and fabrication of various types of drugs, especially nano-based drugs are found to be the most alternative and too cost-effective and environmentally friendly. Among them, metal oxide nanodrugs specially fabricated by green methods are preferred because they enhance the antibacterial action in the presence of various green alternative templates such as various parts of green plants, bacteria, fungi, and viruses, which can act as supportive agents to control their size and shape [11].

It has been seen that metal oxide nanoparticles having high surface area to volume ratio with fast electron transfer kinetics are around to be the best candidates for decorating the bare electrode surface for the measurement and detection of ascorbic acid levels in various sources [12]. Various metal oxide nanoparticles (NPs) such as ZnO, CuO, Fe_3_O_4_, Ag, Cu, Co_3_O_4_, TiO_2_, MgO, and MnO_2_ were synthesized by various methods and used as chemical sensors, biosensors, and gas sensors in the field of industries, environment, food, and drinking items [13–18]. The biogenic processes involve plant components (root, stem, root, peel, leaf, flower, bark, and fruit), spices, fungi, bacteria, yeast, and viruses.

However, physical and chemical synthesis protocols have numerous limitations, such as the use of toxic and expensive capping and reducing agents, high energy consumption, high pressure, and use of nongreen solvents and reagents, so these methods are not simple and require advanced techniques [19]. Moreover, the use of toxic and expensive chemicals as reducing and capping agents resulted in the production of larger particle size, particles having heterogeneous morphology and surface, which is not suitable for the desired applications. As a result, the biogenic approach becomes the most interesting way to fabricate various types of NPs with diversified roles in different fields. Among the biogenic approaches, the use of different parts of green plants extracted as a capping and reducing agent to control the overgrowth of metal oxide nanoparticles is the most favorable synthesis method as compared to the counter parts. Among the different types of metal oxide NPs, cobalt oxide (Co_3_O_4_) NPs received greater significance due to their high redox chemistry, high electrocatalytic activity, fast electron transfer kinetics, efficient stability, and low cost [20].

The plant potato scientifically known as *Solanum tuberosum* is one of the most commonly cultivated food source plants belonging to the family of Solanaceae [21]. Throughout the world, *Solanum tuberosum* is highly used as a common source of food. As the plant is very rich in bioactive molecules that have body building and health keeping function, it is highly cultivated and the increased demand for processed potato products generates large amounts of byproducts from a variety of sources such as peel, leaves, and stems [22]. *Solanum tuberosum* leaf is a useful source of diverse bioactive compounds and well known by its high level of starch, crude fiber, vitamins, amino acids, minerals, acid-soluble and acid insoluble lignin, and lipids [20, 21]. Due this fact, the plant parts, specifically the leaf could be accessed with zero cost since they exist as byproduct and are employed for the biogenic synthesis of various types of NPs, instead of using toxic and too costly capping and reducing agent conductive polymers and chemicals.

In the past, the concentrations and levels of AA and CA in various sources, particularly in diets, have been identified and measured using various commercially and chemically synthesized materials and NPs, but these are not effective and sensitive and selective [17]. *Solanum tuberosum* plant was used for the synthesis of few metal oxides in the past, but no study was reported on CO_3_O_4_ NPs. Thus, we used this plant to synthesise CO_3_O_4_ NPs and studied their multifunctional applications. However, the synthesis of Co_3_O_4_ NPs in the presence of different volume ratios of leaf extract suspension of *Solanum tuberosum* as a capping and reducing agent has not yet been reported. Also, Co_3_O_4_ NPs synthesized using *Solanum tuberosum* plant leaf extract for the sensing of AA and CA in various diets have not yet been reported. Moreover, previous reports have shown that Co_3_O_4_ NPs were prepared by different protocols and their antibacterial potential was investigated on Gram-negative and Gram-positive bacteria species. Although Co_3_O_4_ NPs were fabricated via various chemical and green techniques, there is no scientific document proving the effect of the volume ratios of Co_3_O_4_ NPs on antibacterial activity. The current study focuses on the biogenic synthesis of Co_3_O_4_ NPs using cobalt nitrate hexahydrate precursor in different volume ratios with the suspension of S*olanum tuberosum* leaf as a reducing and capping agent to make this method as a green synthesis approach. The synthesized Co_3_O_4_ NPs are characterized by various techniques to investigate their sensing potential towards AA and CA and also the effect of the volume ratios of the extract and the precursor salt on the sensing potential of AA and CA. Moreover, this work also describes the effect of volume ratios on average crystalline size, morphology, optical property, particle size, and the antibacterial activity against Gram-positive (*S. pyogenes* and *S. aureus)* and Gram-negative (*P. aeruginosa* and *E. coli*).

## 2. Experimental Section

### 2.1. Chemicals and Regents

The necessary chemicals, solvents, and used reagents were ethanol (99.9%, LabTech Chemicals), cobalt nitrate hexahydrate, acetone, dimethyl sulfoxide, Müller-Hinton agar, and sodium hydroxide (Sigma Aldrich). All the chemicals and reagents were of analytical grade, and they were utilized without further purifications.

### 2.2. *Solanum tuberosum* Leaf Preparation and Extraction

The fresh and healthy leaves of S*olanum tuberosum* were collected from the local area without any cost. Later, the collected leaves were washed several times using the distilled water to clean the surface and remove dust and various contaminants. The cleaned leaves of S*olanum tuberosum* were allowed to shadow dry till all the moisture content was completely removed and ready for grinding. The dried leaves were ground using a plant grinding machine followed by packing within a glass bottle covered with aluminum foil [22, 23]. The extraction process was carried out within a 1000 mL volumetric flask by taking 33 g of leaf powder, followed by addition of 450 mL of distilled water. The resulting components were covered with aluminum foil to avoid the effect of light and boiled at 75°C for about 45 minutes. After that, the suspension was cooled to room temperature and filtered using the section filtration glass. Finally, the filtrate was stored packed with a glass bottle covered with aluminum foil and placed within a refrigerator at 4°C for further use.

### 2.3. *Solanum tuberosum* Leaf Templated Biogenic Synthesis of Co_3_O_4_ NPs

The biogenic synthesis of Co_3_O_4_ NPs within various volume ratios were performed using Co(NO_3_)_2_.6H_2_O precursor salt and the extract of *Solanum tuberosum* leaf as a reducing and capping agent. The synthesis process was carried out using 0.25 M of cobalt nitrate hexahydrate and leaf extract of *Solanum tuberosum* within 1 : 1 (50 mL of precursor: 50 mL of extract), 1 : 2 (33.3 mL of precursor: 66.7 mL of extract), and 2 : 1 (66.7 mL of precursor: 33.3 mL of extract) ratios using a separate Erlenmeyer flask. Each Erlenmeyer flask containing two components was placed on a magnetic stirrer and stirred for about 4 hours at room temperature. Later, the pH of the suspensions was monitored using the pH meter, and 15 mL of 1 M NaOH was added as a precipitating agent followed by stirring each of the individual ratios containing the two components for about 20 minutes to maintain the homogenization of the added base. After completion of the reaction, each of the individually formed suspension was placed within a dark area overnight. The formed and settled precipitate was washed three times using absolute ethanol and distilled water via centrifugation at 4,000 rpm. Each volume ratio of the precipitates was collected using a crucible ceramic dish followed by drying at 60°C till all the solvents and the reagents are completely removed followed by calcination using a muffle furnace at 500°C for three hours [24, 25].  Figure 1 shows the schematic of biogenic synthesis of Co_3_O_4_ NPs by employing extract of *Solanum tuberosum* leaf.

### 2.4. Fabrication of Co_3_O_4_ NPs Modified Working Electrode for AA and CA Sensing

The preparation of carbon paste and modified carbon paste working electrode (CPWE) was performed by using graphite powder having approximated 33 *μ*m sizes. In order to improve the strength and also the viscosity behavior of the electrode, silicone oil reagent was used. Then, the biogenic-synthesized Co_3_O_4_ NPs were formed within 1 : 1, 1 : 2, and 2 : 1; each of the three ratios were mixed separately with the graphite powder and the silicon oil reagent followed by grinding using mortar and pestle till the mixed components becomes completely homogenized. The formed paste was then packed within the Teflon tube, with the presence of efficient pressure to ensure enough electrical contact with the presence of copper wire. The surface of the modified generated CPWE was generated rapidly by extruding a small plug of the prepared paste followed by smoothing the resulting obtained surface on wax paper until the surface becomes shiny enough [26, 27]. Finally, the biogenic-synthesized Co_3_O_4_ (1 : 1) NPs, Co_3_O_4_ (1 : 2) NPs, and Co_3_O_4_ (2 : 1) NPs were employed as green alternative and cost-effective working electrodes by modifying the bare CPWE for the sensing of AA and CA. Here, Ag/AgCl and KCl were used as reference and counter electrodes, respectively.

### 2.5. Antibacterial Analysis

The antibacterial performance of the various green-synthesized Co_3_O_4_ NPs was investigated against Gram-positive (*S. pyogenes* and *S. aureus*) and Gram-negative (*P. aeruginosa* and *E. coli*) species via the disc diffusion method. Initially, the sufficient amount of nutrient broth agar was prepared in 100 mL distilled water, and then after, it was subjected to sterilization. The prepared cultures were inoculated in nutrient broth and were kept on a rotary shaker at 35°C ± 2°C for 24 h at 160 rpm. Ampicillin and DMSO were used as positive control/standard and solvent, respectively. Then, the nutrient agar was prepared within 100 mL distilled water using 6 g nutrient agar and 0.8 g agar-agar followed by well shaking till it became uniformly homogenized. The plates were then inoculated by dipping a sterile cotton wool swab into the resulting suspension followed by complete drying. Then, the plates were incubated at 37°C for about 24 h and checked for the zone of inhibition [27].

### 2.6. Characterization Techniques

The formation of Co_3_O_4_ NPs and the role of the extract were confirmed by various characterization techniques. The crystallinity, average crystalline size, and purity of the synthesized NPs were explored by using an X-ray diffractometer (XRD-7000, Shimadzu Co., Japan), and XRD patterns were recorded in the 10–80^o^ 2*θ* range using CuK*α* (=1.54056Å) radiation operated at 40 kV and 30 mA. The structural morphology of each of the ratios of the biogenic-synthesized Co_3_O_4_ NPs were confirmed using SEM equipped with energy dispersive spectroscopy (SEM-EDX-EVO 18 model-ALTO 1000 Cryo attachment). The particle size, crystallinity nature, and morphology of the synthesized Co_3_O_4_ NPs were also checked via transmission electron microscopy such as TEM, HTREM, and SAED pattern (TEM, JEOL TEM 2100 HRTEM). The role of the extract used during the synthesis process was confirmed using Fourier transform spectroscopy (PerkinElmer 65). The optical behavior was studied by diffuse reflectance spectroscopy in the range between 200 and 800 nm using the Shimadzu UV-Vis1800 double beam spectrophotometer (Shimadzu, Tokyo, Japan). Investigation of electrochemical properties was carried out using cyclic voltammetry on a CHI608E potentiostat (CH Instruments, Inc., Austin, TX, USA) in the presence of the three electrodes and KOH as an electrolyte.

## 3. Results and Discussion

### 3.1. XRD Analysis

The crystallographic nature of the biogenically synthesized Co_3_O_4_ NPs within various volume ratios was characterized by XRD.  Figure 2 shows the resulted XRD pattern of Co_3_O_4_ NPs and the diffraction peaks were observed at 2*θ* values of 19.01°, 31.37°, 36.85°, 38.5°, 44.88°, 55.71°, 59.4°, 65.26°, 74.31°, and 77.5° corresponding to the Miller indices (hkl) value of (111), (220), (311), (222), (400), (422), (511), (440), (533), and (622), respectively. The diffraction peaks of Co_3_O_4_ NPs were found to be in a good agreement with JCPDS card number 042–1467 [28], which confirms the formation of pure Co_3_O_4_ NPs without the formation of any secondary phase. The calculated average crystalline sizes were estimated to be 25.83, 21.05, and 27.98 nm for the volume ratios of 1 : 2, 1 : 1, and 2 : 1, respectively. It has been observed that, among the three volume ratios, Co_3_O_4_ (1 : 1) NPs possess smaller average crystalline size as compared to the remaining ratios. This might be due to the greater amount of the leaf suspension used during the synthesis process, which results in higher proportions of capping and stabilizing agents; this in turn effectively stabilizes the synthesized Co_3_O_4_ (1 : 1) NPs [15, 28].

As can be observed from the XRD spectra, the peak heights of Co_3_O_4_ (2 : 1) NPs are too great as compared to the counter parts, and this is in agreement with its relatively large average crystalline size, and this might be due to the use of smaller volume of leaf extract. Moreover, the XRD graph for each of the various ratios was found to be in good agreement with the literature report before [15, 24, 25], which indicates that pure Co_3_O_4_ NPs are formed from the reaction between cobalt nitrate hexahydrate and extract of *Solanum tuberosum* leaf.

### 3.2. Morphology Analysis Using SEM

Figures 3(a)–3(c) show the corresponding SEM morphology of Co_3_O_4_ (1 : 2), Co_3_O_4_ (1 : 1), and Co_3_O_4_ (2 : 1), respectively. It has been observed that the morphologies of Co_3_O_4_ (1 : 1) and Co_3_O_4_ (2 : 1) NPs are relatively more homogenized compared to the remaining ratios. The SEM analysis result also confirms that all the three ratios of Co_3_O_4_ NPs possess nearly spherical structural morphology. In addition to this, the synthesized Co_3_O_4_ NPs also showed honeycomb-like structure. It is clearly observed from the SEM image that all the ratios of Co_3_O_4_ NPs are too crystalline. In addition, Co_3_O_4_ NPs are scattered over the surface without any aggregated particles; this might be highly contributed due to the presence of bioactive molecules from the leaf [29, 30].

Figures 3(a)–3(c) show the EDX result analysis of Co_3_O_4_ (1 : 2), Co_3_O_4_ (1 : 1), and Co_3_O_4_ (2 : 1) NPs. The results confirm that the Co_3_O_4_ NPs contain Co and O as major elements. Furthermore, the EDX also confirms the existence of K and Zn additional minor peaks in trace amount, which might be contributed and occurred due to the usage of the standard and also during the preparation of the sample for SEM-EDX analysis [30].

### 3.3. TEM and SAED Analysis

In order to investigate and gather additional information related to in-depth morphological features of Co_3_O_4_ (1 : 1) NPs, samples were characterized via TEM (50 and 20 nm magnifications), SAED, and HRTEM techniques and are shown in Figure 4.

Figures 4(a) and 4(b) show the TEM images of the Co_3_O_4_ NPs (1 : 1) at 50 and 20 nm scale magnification, respectively. The morphology was found to be spherical as confirmed by SEM analysis too. Assembled spheres indicated the presence of good connectivity, dispersibility, and homogeneity between the formed particles. Moreover, Figure 4(c) shows the SAED pattern and the polycrystalline nature of the S*olanum tuberosum* leaf extract mediated synthesized Co_3_O_4_ NPs. The white circular spots in the center of the SAED image correlated to the (111), (220), (311), and (222) and (400) lattice planes, which well matched with the obtained XRD results. As shown in Figure 4(d), the major lattice plane (311) was calculated to be 0.25 nm and found to fit with the fringe spacing value, which is in good agreement with the previously reported work [31] and well agreed with the XRD value of 2*θ* with 36.10. Figure 4(d) of HRTEM image also confirms the polynanocrystalline nature of Co_3_O_4_ (1 : 1), and it has well-defined shape and visible grain boundaries, which can be achieved via a controlled synthesis procedure in the presence of bioactive molecules from the crude extract of *Solanum tuberosum* leaves. Furthermore, Figures 4(e) and 4(f) with the IFFT magnified (Figure 4(g)) image was the output of the lattice fringe analysis, and again, the d-spacing value of 0.31 nm is found to be well matched with the second major peak presented under the XRD data at (220) having 2*θ* with 31.00. The presence of stacking-like faults on the surface of the *Solanum tuberosum* leaf extract templated Co_3_O_4_ (1 : 1) NPs suggests and inputs an insight about the nanopolycrystalline nature, as shown in Figure 4(g).

### 3.4. Functional Group Analysis

FTIR analysis (Figure 5) for the biogenically synthesized, calcined (a) and uncalcined (b) Co_3_O_4_ (1 : 1) NPs and the leaf extract of *Solanum tuberosum* (c) were carried out in order to explore the formation of Co_3_O_4_ NPs and confirm the functional groups present in the leaf extract. This in turn enables to identify the bioactive molecules which were actively involved during the synthesis process as stabilizing and capping agents to prevent the overall growth of Co_3_O_4_ NPs [32]. Figure 5 shows the FTIR spectra of calcined and uncalcined Co_3_O_4_ NPs and leaf extract of *Solanum tuberosum* and were recorded in the range of 4000–400 cm^−1^.

The broad peak observed in the spectrum at around 3426 cm^−1^ represents the O-H stretching with a C = O peak, confirming aliphatic carboxylic acid. While, the prominent levels of absorption peak located at around 2911 cm^−1^ reveal the presence of C-H stretching vibrations of an aromatic aldehyde. The peak observed around 2322 cm^−1^ represents the amide (C ≡ N) functional groups [33]. The medium absorption peak observed at 1638 cm^−1^ corresponds to C = O peak, which indicates the ketone functional group and also the ammine functional group. The band observed at 1422 cm^−1^ corresponds to C-C stretching of the aromatic groups obtained from the leaf extract of *Solanum tuberosum*. An absorption peak found at 1056 cm^−1^ corresponds to the saturated primary alcohol containing the C-O bond. The narrow peak observed around 504 cm^−1^ indicates the formation of Co-O stretching. The same phenomenon was observed in the case of both the uncalcined and leaf extract; the only difference is the slight shift in the location of the peaks. This again confirms that the extract has played a great role to prevent the overgrowth of Co_3_O_4_ NPs during the synthesis process [33–35]. It is possible to elucidate the formation of Co_3_O_4_ NPs with many surface hydroxyl function groups.

### 3.5. UV-DRS Analysis

The optical absorption properties and band gap energy of *Solanum tuberosum* leaf extract templated synthesized Co_3_O_4_ NPs have been investigated by characterizing via UV-Vis spectroscopy. As shown in Figure 6(a), the absorption spectra of the green templated Co_3_O_4_ NPs were characterized in the range of 200–800 nm. It has been found that each of the three volume ratios of Co_3_O_4_ NPs showed two absorption peaks, which is found within the range of 265–360 nm and 400–610 nm. In all of the ratios, the first absorption peaks depict the charge transfer process of O^2−^ into Co^2+^, while the latter peak presents the resulting charge transfer of O^2−^ into Co^3+^. Those absorption peaks in turn showed the formation of green p-type Co_3_O_4_ NPs [34].

Furthermore, Figure 6(b) shows Tauc plot of *Solanum tuberosum* leaf templated Co_3_O_4_ NPs. The energy band gaps were deduced to be 1.83, 1.77, and 2.19 eV for the volume ratios of 1 : 1, 1 : 2, and 2 : 1, respectively. Among the three volume ratios of Co_3_O_4_ NPs, 2 : 1 volume ratio has larger band gap energy and so possesses high quantum confinement as compared to the counter parts. The band gap energy analysis confirmed the formation of stable Co_3_O_4_ NPs, as also supported by the previous reports [35].

### 3.6. CV and EIS Studies of Co_3_O_4_ NPs

The electrochemical properties of the synthesized Co_3_O_4_ NPs within various volume ratios in the presence of *Solanum tuberosum* leaf extract as biotemplated were investigated via CV, EIS, and amperometry techniques. Figures 7(a)–7(c) supported with Table 1 show the CV plots of Co_3_O_4_ (1 : 2, 1 : 1, and 2 : 1 volume ratios) green-synthesized nanoelectrodes at various scan rates, respectively. In three of the green-formed Co_3_O_4_ nanoelectrodes, it has been observed that the cathodic peak increases with increasing of scan rate, and these twists were found to be asymmetric quasirectangular in shape. The reversibility of Co_3_O_4_ (1 : 1) nanoelectrodes is relatively fast compared to the remaining two ratios of Co_3_O_4_ nanoelectrodes because of least *E*_*O*_−*E*_*R*_ value (0.178°v) [36], which can be attributed due to the smaller average crystallite size, and this intern indicates the high catalytic behavior of Co_3_O_4_ (1 : 1) green nanoelectrodes which is one pillar criteria for the sensing of AA and CA [37].

Moreover, for further characterization and investigation of Co_3_O_4_ nanoelectrodes, the interfacial properties were analyzed using the EIS technique, which could be used to clarify the impedance changes in the electrode modification process.

It has been noted that the green-synthesized Co_3_O_4_ nanoelectrodes exhibited almost vertical linearity, which makes an approximate angle of 90° in presence of real axis, noted at the frequency level which might vary from low to high frequency region. As shown in Figure 8, Co_3_O_4_ (1 : 1) nanoelectrodes showed the ideal ion diffusion behavior due to its homogenized surface morphology and smaller average crystallite size, as can be confirmed from the XRD and SEM analyses. In all of the three volume ratios of the green nanoelectrodes, the resulting impedance originates due to the frequency-dependent ideal ion diffusion at the interface of the green nanoelectrodes and basic electrolyte solution [11, 38, 39].

In addition to the CV and EIS characterization techniques, the green Co_3_O_4_ nanoelectrodes were also subjected to amperometry analysis in order to confirm the sensitivity, limit of detection, and also the linear range of Co_3_O_4_ nanoelectrodes; which was used for the preparation of GCPE and then for the sensing of both AA and CA in the presence of basic electrolyte. All of the green-fabricated Co_3_O_4_ nanoelectrodes showed improved current response (Figure 9). However, among three green nanoelectrodes, Co_3_O_4_ (1 : 1 and 2 : 1) nanoelectrodes presented best current response due to their uniform homogenized surface structure and small average crystalline size and enhanced catalytic activity, which might be contributed due to the use of smaller volume of the extract during the synthesis process [40].

Figures 10(a)–10(c) show CA sensing potential of green-synthesized Co_3_O_4_ NPs fabricated using the 1 : 2, 1 : 1, and 2 : 1 volume ratio modified CPE. As shown in Figures 10(a)–10(c), as the concentration of CA increases, the resulting current also increases, and at high CA concentration, the current response reaches saturated point. This suggests that the active surface sites of NPs are saturated with CA molecules, which proves that the response was a surface process, and this in turn is an indication of the high electrocatalytic activity of the fabricated nanoelectrodes.

The 1 : 1 and 2 : 1 volume ratio modified CPWE shows better detection potential as compared to the 1 : 2 volume ratio fabricated modified CPWE [41]. This might be contributed due to the better electron transfer kinetics, which could be contributed to the more homogenized surface area and high catalytic behavior.

Figure 11 shows the electrochemical sensing of AA using the various volume ratio of Co_3_O_4_ NPs-modified CPWE. In the same manner, as the concentration of acetic acid is enhanced, the current response also improved, which suggests the high catalytic behavior of the green-fabricated Co_3_O_4_ nanoelectrodes.

It has been found that the 1 : 2 and 1 : 1 volume ratios of Co_3_O_4_ NPs-modified CPWE showed better sensing of ascorbic acid at a lower potential. This is possibly due to the smaller average crystallite size as can be obtained from the XRD analysis, which provides high surface area, and this suggests that the electron transfer kinetics also improved. Moreover, Figures 10(a) and 10(b) show the better detection capability of the 1 : 2 and 1 : 1 volume ratios at a lower potential as compared to the counter parts [42].

### 3.7. Antibacterial Activity

The antibacterial activity of *Solanum tuberosum* leaf extract templated synthesized Co_3_O_4_ NPs was investigated via the method of disk diffusion. As shown in Figure 11 and supported by Table 2, the antibacterial activity of each of the volume ratios of Co_3_O_4_ NPs was enhanced with increasing the concentration of the nanoparticles. The antibacterial activity of Co_3_O_4_ (1 : 1) nanoantibiotics was found in the range between 8 and 12.5 mm against *S. pyogenes, S. aureus, P. aeruginosa*, and *E. coli*. While, the antibacterial activity of Co_3_O_4_ (2 : 1) nanoantibiotics showed zone of inhibition in the range of 7–11 mm against the selected bacteria. In addition to those, the antibacterial zone of inhibition for the Co_3_O_4_ (1 : 2) nanoantibiotics was measured in the range of 10–16 mm. The antibacterial activity for the three volume ratios was found to be enhanced with an increasing amount of the leaf extract of the template. As shown in Figure 12 and Table 2, green Co_3_O_4_ (1 : 2) nanodrugs were found to be the most efficient and effective antibiotics as compared to the counter parts. This high antibacterial performance of green Co_3_O_4_ (1 : 2) nanoantibiotics might be contributed due to the high ROS production. In turn, the high ROS production results from the use of large volume of *Solanum tuberosum* leaf extract [9]. Furthermore, the antibacterial activity of Co_3_O_4_ (1 : 1) green nanodrug showed enhanced performance next to 1 : 2 volume ratios. While, the 2 : 1 volume ratio of Co_3_O_4_ nanodrugs showed less performance as compared to the two volume ratios of Co_3_O_4_ nanodrugs.

Green-synthesized Co_3_O_4_ nanodrugs were found to be a promising cost-effective antibiotics against the Gram-positive bacteria as compared to Gram-negative bacteria. Since, Gram-negative bacteria species contain double cell membrane, which prevents the entry of the nanodrugs into the cell wall of those bacteria [43–45]. Table 2 provides the summery of zone of inhibition of Co_3_O_4_ nanodrugs at a concentration of 50, 75, and 100 mg/mL against *E. coli*, *S. aureus*, *P. aeruginosa*, and *S. pyogenes*.

From Table 2, it can be found that all of the various volume ratios of Co_3_O_4_ nanodrugs present enhanced activity against Gram-positive bacteria with an increasing concentration of the drug.

## 4. Conclusion

In the present findings, Co_3_O_4_ NPs were successfully synthesized within various volume ratios in the presence of *Solanum tuberosum* leaf extract as a green alternative template. In order to explore the optical, electrocatalytic, and surface plasmon characteristics, the green-synthesized Co_3_O_4_ NPs were characterized using XRD, SEM, EDX, TEM, HRTEM, SAED, FTIR, and UV-DRS. Moreover, the synthesized NPs were used as green alternative and cost-effective nanoelectrodes for the detection of CA and ascorbic acid. The XRD analysis reveals the average crystallite sizes of 25.83, 21.05, and 27.98 nm for the volume ratios of 1 : 2, 1 : 1, and 2 : 1 Co_3_O_4_ NPs, respectively. SEM-EDX and TEM including HRTEM and SAED indicates that the green-synthesized Co_3_O_4_ NPs were too crystalline having spherical structure without any secondary phase and foreign materials. In addition, the FTIR analysis confirms the role of leaf extract of *Solanum tuberosum* as both capping and reducing agents that prevent the overgrowth of Co_3_O_4_ NPs and also indicates the formation of Co-O stretching. The UV-DRS result suggests the energy band gap for Co_3_O_4_ NPs synthesized with the volume ratio of 1 : 2, 1 : 1, and 2 : 1 was deduced to be 1.77, 1.83, and 2.19 eV, respectively. The sensing performance of the green-synthesized Co_3_O_4_ nanoelectrodes was found to be good towards AA and CA. It has been found that the green-synthesized Co_3_O_4_ nanoelectrodes were effective for both AA and CA. At the end, the antibacterial activity of the various volume ratios of green-synthesized Co_3_O_4_ NPs was evaluated against *S. pyogenes*, *S. aureus*, *P. aeruginosa*, and *E. coli*. Of the three volume ratios, the 1 : 2 ratios showed enhanced antibacterial activity (16 mm) as compared to the other counter parts.

## Figures and Tables

**Figure 1:** Diagrammatical biogenic synthesis of Co_3_O_4_ (1 : 1) NPs.

**Figure 2:** XRD pattern of *Solanum tuberosum* leaf templated Co_3_O_4_ NPs.

**Figure 3:** SEM images of *Solanum tuberosum* leaf templated formed Co_3_O_4_ NPs within (a) 1 : 2, (b) 1 : 1, and (c) 2 : 1 ratio with their corresponding EDX.

**Figure 4:** TEM micrograph of Co_3_O_4_ (1 : 1) NPs at (a) 50 nm and (b) 20 nm magnification, (c) SAED pattern, (d) HRTEM image (1), (e) HRTEM image (2), ((f) HRTEM image (3), and (g) the magnified IFFT profile.

**Figure 5:** FTIR spectra of (a) calcined Co_3_O_4_ (1 : 1) NPs, (b) uncalcined Co_3_O_4_ (1 : 1) NPs, and (c) *Solanum tuberosum* leaf extract.

**Figure 6:** DRS spectra of green-synthesized Co_3_O_4_ NPs (a) and their corresponding band gap energy (b).

**Figure 7:** CV plots of *Solanum tuberosum* leaf extract templated synthesized Co_3_O_4_ NPs electrode. (a) CV plots of *Solanum tuberosum* leaf extract templated synthesized Co_3_O_4_ (1:2) NPs electrode. (b) CV plots of *Solanum tuberosum* leaf extract templated synthesized Co_3_O_4_ (1:1) NPs electrode. (c) CV plots of *Solanum tuberosum* leaf extract templated synthesized Co_3_O_4_ (2:1) NPs electrode.

**Figure 8:** EIS spectra of green-synthesized Co_3_O_4_ nanoelectrodes.

**Figure 9:** Amperometry response of Co_3_O_4_ nanoelectrodes at various volume ratios.

**Figure 10:** CV plots of Co_3_O_4_ ((a) 1 : 2, (b) 1 : 1, and (c) 2 : 1) modified CPWE CA sensor.

**Figure 11:** CV plots of Co_3_O_4_ ((a) 1 : 2, (b) 1 : 1, and (c) 2 : 1 volume ratios) modified CPWE ascorbic acid sensor.

**Figure 12:** Zone of inhibition of green Co_3_O_4_ (1 : 2, 1 : 1, and 2 : 1) nanodrugs against *E. coli*, *S. aureus*, *P aeruginosa*, and *S. pyogenes* at 50, 75, and 100 mg/mL concentration.

**Table 1:** The CV and EIS result for Co_3_O_4_.

Co_3_O_4_ NPs	*E*_*O*_ (V)	*E*_*R*_ (V)	*E*_*O*_−*E*_*R*_ (V)

1 : 2	0.234	0.031	0.203
1 : 1	0.222	0.044	0.178
2 : 1	0.238	0.029	0.209

**Table 2:** The zone of inhibition of Co_3_O_4_ nanodrugs against *E. coli*, *S. aureus*, *P. aeruginosa*, and *S. pyogenes.*

Ratio	Concentration (mg/mL)	Bacterial species and zone of inhibition (mm)			
		*E. coli* ATCC25922	*S. aureus* ATCC25923	*P. aeruginosa* ATCC27853	*S. pyogenes* ATCC19615

1 : 1	50	9	9	8	9
	75	10	11	9	10
	100	11.5	12.5	11	12

2 : 1	50	7	8	7	8
	75	9	9	8.5	9
	100	10	11	9	10

1 : 2	50	11	12	10	11
	75	13	14	12	12
	100	15	16	14	15
Ampicillin		14	15	13.5	14.5

## Data Availability

The data used to support the findings of this study are included within the article.
